RETRACTED

# Liraglutide Is Protective against Brain Injury in Mice with Febrile Seizures by Inhibiting Inflammatory Factors

**DOI:** 10.1155/2022/7563281

**Published:** 2022-04-29

**Authors:** Xing Wang, Fei Yang, Liling Deng, Di Qiu, Yao Liu, Yang Kang

**Affiliations:** Department of Pediatrics, The Third Affiliated Hospital of Qiqihar Medical University, Qiqihar 161000, China

## Abstract

The febrile seizure (FS) is a common disease in emergency pediatrics, and about 30% of patients are children aged between 6 months and 5 years. Therefore, we aim to observe the protective impact of liraglutide (LIR) on brain injury in mice with FS and to explore its relevant mechanisms. Male SD mice were selected, and the FS model was established by heat bath method. The behavioral score was performed on mice with Racine grading, and nerve cells in apoptosis in the hippocampus were determined by TUNEL. The content of glutamate was determined by ELISA. mRNA levels and protein expression of GLP-1, GLP-1R, IL-1*β*, IL-6, TNF-*α*, and cleaved-caspase 3 were examined in mice by q-PCR and WB. Protein expression of *γ*-aminobutyric acid was influenced by WB as well. LIR prolonged the seizure latency and seizure duration in mice with FS. The GLP-1 and GLP-1R in the mouse hippocampus with FS expressed highly and also inhibited the number of nerve cells in apoptosis, decreased glutamate content, and increased *γ*-aminobutyric acid expression in the mouse hippocampus with FS. In addition, The IL-1*β*, IL-6, and TNF-*α*, in the mouse hippocampus with FS expressed to reduce with LIR. LIR is protective against brain injury in mice with FS and protects brain injury by inhibiting inflammatory factors in mice with FS. Our finding provides a reference for mitigating and delaying the development of FS as well as the prevention and treatment of brain injury caused by FS.

## 1. Introduction

Febrile seizures (FS) are a prevalent type of seizures in children aged between 6 months and 5 years [1, 2]. There is a lot of evidence to show that inflammation is closely connected to the pathogenesis of FS [3, 4]. There is a close relationship between interleukin 6 (IL-6) levels in plasma and the growth of FS [5]. Interleukin 1*β* (IL-1*β*) is an important neuroimmune mediator and contributes to the development of FS [6]. The levels of IL-6, IL-1*β*, and TNF-*α* are remarkably improved [7]. The release of IL-1*β* is relevant to the type 1 receptor (IL-1RI) that is expressed by neurons in the hippocampus, resulting in an increase in neuronal excitability and decreasing seizure threshold. IL-1*β* receptor-deficient mice can inhibit the production of FS in mice. It can cause brain injury by rising the functions of extracellular excitatory amino acids, like glutamate and inhibiting the functions of *γ*-aminobutyric acid receptors. TNF-*α* released from reactive astrocytes and activated microglia can promote the release of glutamate [8] and regulate the firing of neurons and seizures. Thus, it is essential to control the severity of neuroinflammation for preventing FS.

RETRACTED

Glucagon-like peptide 1 (GLP-1), as a glycaemic hormone, is important for blood glucose control and weight regulation [9]. Liraglutide (LIR) acts in the body by binding to GLP-1R, as an analogue of GLP-1, which has a significant impact on the treatment of diabetes mellitus (DM) [10]. LIR is protective against neurons in different models of brain diseases [11].

GLP-1 analogue is antiepileptic in the pentamethazol (PTZ) model, and the mice that lack GLP-1R exhibited lighter seizure thresholds [12]. LIR is protective in a few models of seizures epilepsy characterized by neurodegeneration. Moreover, it has been shown that the GLP-1/GLP-1R signaling pathway participates in FS pathogeny, whereas the specific mechanism of action has not been defined [13]. Studies have shown the potential antiepileptic impacts on LIR in different mouse models [14]. These findings have shown that in a few models of convulsant epilepsy characterized by neurodegeneration, LIR could be a viable new strategy for preventing and treating epileptogenesis and it had a relationship with behavior and the change of cognition.

There are many preclinical studies confirming that GLP-1/GLP-1R signaling can significantly reduce the inflammation in multiple parts of the body, such as the gut, lung, endothelial cells, and central nervous system (CNS) [15]. The expression of inflammatory factors increased the secretion of GLP-1 rapidly, especially IL-6 [16], however, the proinflammatory cytokine, TNF-*α* expressed lower with GLP-1 [17]. It was found that the effect of protection of GLP-1 analog, exendin-4, on neural cells is connected with the decreased mRNA expression of proinflammatory factors, like IL-17, IL-1*β*, IL-6, and TNF-*α*, and exendin-4 has effects on mRNA of IL-1*β* and TNF-*α* in lipopolysaccharide- (LPS-) induced microglia. It suggests that GLP-1 may be a regulator of the inflammation of CNS. Thus, it is hypothesized that LIR may be protective against brain injury in FS by inhibiting inflammatory factors in the body.

Therefore, we observed the protective impact of liraglutide (LIR) on brain injury in mice with FS. And we adopted behavioral score on mice with Racine grading and determined nerve cells in hippocampus by TUNEL.

## 2. Experimental Methods

### 2.1. Research Object

Thirty 14-day SPF male SD mice, obtained from the Model Animal Research Center of Nanjing University, were randomized into the control, FS, and FS+LIR groups (*n* = 10 per group). The mouse FS model was established by a repeated hot water bath (at 44.5°C for 5 min), once every other day for 10 times in total. Meanwhile, mice in the FS+LIR group were subcutaneously injected with LIR at 0.3 mg/(kg·d), and the control and FS groups were given equal amounts of saline for 20 days.

RETRACTED

Racine grading was performed on mice for behavioral scores, to record the seizures latency and seizure duration in mice: level 0: normal behavior; level 1: seizures of ear and face; level 2: loss of postural control; level 3: myoclonic seizures and rearing; level 4: clonic seizures, mice lying aside; and level 5: repeated severe tonic-clonic seizures.

### 2.2. TUNEL Staining

Mice's hippocampi were preserved in 4% paraformaldehyde, embedded in paraffin wax, and then diced up (with the thickness of 4 *μ*m). Then, the slides were dewaxed in xylene and hydrated with an ethanol gradient. Apoptosis in hippocampal neurons of mice was detected with TUNEL (terminal deoxynucleotide transferase-mediated detection of dUTP notch terminal markers) staining kit (KeyGEN BioTECH, China). TdT and dUTP were mixed in the kit in a ratio of 1 : 9 and dropped on glass slides. After TUNEL labeling, hippocampal neurons were stained with DAPI to detect nucleus. TUNEL-positive cells labeled with a green fluorescent protein in the hippocampus were visualized by fluorescence microscopy. Subsequently, three microscopy fields were randomly selected in the hippocampus and TUNEL-positive cells were counted blindly to calculate the percentage of TUNEL-positive cells in total cells.

### 2.3. q-PCR

mRNA of GLP-1, GLP-1R, IL-1*β*, IL-6, and TNF-*α* were examined in the mouse hippocampus. High fever is the initiating factor of FS, which essentially involves inflammation, and IL-1*β* is a key component of inducing FS. Furthermore, it was found that levels of IL-1*β* were remarkably increased in hippocampus of epileptic animals [18]. Fresh hippocampus was ground into homogenates, after which total RNA was isolated from tissues according to the total RNA extraction kit's instructions (Solebo, China). And then, cDNA was synthesized by reverse transcription of RNA and amplified by qPCR with SYBR Green (Baori Medical Technology Co., Ltd., China). Primer sequence is as follows (Shanghai Sangon, China):

GLP-1: forward 5′-CAGAAGTTGGTCGTGAGGCA-3′, reverse 5′-AGCCTTTCACCAGCCAAGCAA-3′; GLP-1R: forward: 5′-GTTGAGGGGGAGTTTGGA-3′, reverse: 5′-ACCCCAAAAATAAAACCTCCAACTCTA-′; IL-1*β*: forward 5′-TACCTATGTCTTGCCCGTGG-3′, reverse: 5′-TAGCAGGTCGTCATCATCCC-3′;

IL-6: forward: 5′-CTGCTCTGGTCTTCTGGAGT-3, reverse: 5′-TGGAAGTTGGGG-TAGGAAGG-3';

TNF-*α*: forward: 5′-GGTGATTGGTCCCAACA-3′, reverse: 5′-GTCTTTGAGATCCATGCC-3′; and GAPDH: forward 5′-GGCATTGCTCTCAATGACAA-3′, reverse 5′-ATGTAGGCCATGAGGTCCAC-3′.

RETRACTED

Amplification conditions were 45 cycles, at 95°C for 15 s, at 62°C for 15 s, and at 72°C for 45 s. The information was examined using 2^-*ΔΔ*Ct^, with GAPDH as the inner citation. The multiples of the average value of the control group were used to express the mRNA of various indexes in the mouse hippocampus.

### 2.4. Western Blot

The expression of GLP-1, GLP-1R, IL-1, IL-6, TNF-*α*, cleaved-caspase 3, and *γ*-aminobutyric acid was determined in the hippocampus of mice by Western blot. The fresh hippocampus was collected for adequate grinding, and the BCA assay for the protein concentration. Proteins were diluted with 5x loading buffer for denaturation by boiling for 5 min. The 40 *μ*g protein loading sample was placed onto 10% gradient polyacrylamide gel, transferred to the PVDF membrane by 120 V electrophoresis, and sealed with skim milk powder, incubating primary antibody at 4°C overnight: GLP-1 (1 : 1000, CST), GLP-1R (1 : 500, Abcam), IL-1 (1 : 1000, Abcam), IL-6 (1 : 1000, Abcam), TNF-*α* (1 : 1000, Abcam), cleaved-caspase 3 (1 : 1000, CST), *γ*-aminobutyric acid (1 : 1000, CST), and *β*-actin (1 : 5000, Sigma). The second antibody was cultured for 2 h at room temperature, and ECL solution was dropped for exposure.

### 2.5. ELISA

The protein concentration of glutamate in the hippocampus of mice was determined with the glutamate content ELISA detection kit (Solebao, China). 0.1 g of fresh hippocampus quality was harvested from mice, and the tissue was homogenized by adding 5 mL of reagent. The supernatant was taken away by centrifugation at 8,000 rpm at room temperature for 10 min, and standard curves were made. Reagents were added according to the kit instructions and mixed for 20 min with a 90°C water bath. The microplate detector was preheated for 30 min, and OD A was recorded at the wavelength of 570 nm. Then, we calculated the glutamate content.

### 2.6. Statistical Analysis

Statistical analysis was carried SPSS 24.0 (SPSS, USA). The normal distribution of the data was checked, and all data were expressed as mean ± standard deviation ($\bar{x}\pm s$). After LSD, multiple comparison tests were conducted using the independent sample *T* test and one-way ANOVA. *P* was calculated to be two-sided, and *P* < 0.05 suggests being remarkable statistically.

## 3. Results

### 3.1. Liraglutide Prolonged the Seizure Latency and Seizure Duration in Mice with Febrile Seizures

To investigate the association between LIR and febrile seizures, we induced seizures in mice. Meanwhile, the FS+LIR group was subcutaneously injected with LIR. Mice were scored by Racine grading. The FS group was found to score much higher than the controls. Moreover, the score of the FS group was much higher compared with the FS+LIR group (Figure 1(a)), showing that LIR had a considerable therapeutic impact on FS.

RETRACTED

The seizure latency and seizure duration were also recorded, and prolonged seizure latency was found in the FS+LIR group (Figure 1(b)), and seizure duration was significantly shorter (Figure 1(c)). These results also suggested an obvious therapeutic effect of LIR on FS.

### 3.2. Liraglutide Increased the Expression of GLP-1 and GLP-1R in the Hippocampus of Mice with Febrile Seizures

To further clarify the relevance of LIR and FS, the fresh hippocampus was taken and mRNA of GLP-1 and GLP-1R in the hippocampus of each group were detected. It was found that mRNA of GLP-1 and G LP-1R was significantly reduced in the hippocampus of mice with FS compared with those of the controls. However, mRNA of GLP-1 and G LP-1R significantly increased in the hippocampus of the FS+LIR group (Figures 2(a) and 2(b), *P* < 0.001).

GLP-1 and GLP-1R expressions were examined in the mouse hippocampus with Western blot. Lower GLP-1 and GLP-1R expressions were found in mouse hippocampus with FS, compared with that of the controls. However, the expression of GLP-1 and G LP-1R obviously increased in the FS+LIR group (Figures 2(c)–2(e)).

The above results showed the occurrence of FS in mice is closely related to GLP-1 expression and its receptors.

### 3.3. Liraglutide Inhibited Apoptosis, Decreased Glutamate Content, and Increased *γ*-GABA Expression in Mice with FS

Results 1 and 2 validated a negative correlation between LIR and the development of FS, and we further considered LIR's effect on brain injury of FS. The apoptosis in hippocampal nerve cells was observed with TUNEL, and the result revealed an increased amount of apoptosis in the hippocampus of the FS group than the controls. The quantity of apoptotic neural cells in mice decreased in the hippocampus of the FS+LIR group than in the FS group (Figure 3(a)).

The cleaved-caspase 3 of apoptosis in the hippocampus of mice was detected with Western blot and showed higher cleaved-caspase 3 expression in the FS group than in the controls. However, the protein expression of cleaved-caspase 3 was lower in the hippocampus of the FS+LIR group than in the FS group. The above results suggested that LIR inhibits the apoptosis of nerve cells in hippocampus of mice with FS (Figure 3(c)).

Thereafter, the content of glutamate was detected in the hippocampus of mice. The results showed that glutamate was higher in the FS group than the controls. However, the glutamate content decreased in the hippocampus of the FS+LIR group (Figure 3(d)). And we detected protein expression of *γ*-aminobutyric acid for inhibitory amino acids in the hippocampus. The findings proved that the expression of inhibitory amino acid *γ*-aminobutyric acid was remarkably decreased in the FS group than the controls. However, the expression of *γ*-aminobutyric acid increased in the hippocampus of the FS+LIR group (Figure 3(e)). It suggested that LIR reduces brain injury in mice with FS.

RETRACTED

### 3.4. Liraglutide Inhibited the Expression of Inflammatory Factors in the Hippocampus of Mice with FS

To further explore whether LIR is protective against FS brain injury by inhibiting inflammatory factors within the body, inflammatory factors in the hippocampus of mice were detected.

q-PCR revealed that IL-1*β*, IL-6, and TNF-*α* increased in mice hippocampus in the FS group compared with those of the controls. mRNA of IL-1*β*, IL-6, and TNF-*α* was reduced in the FS+LIR group (Figures 4(a)–4(c)). Western blot showed IL-1*β*, IL-6, and TNF-*α* increased in the FS group than those of the controls. Protein expression of IL-1*β*, IL-6, and TNF-*α* was reduced in the FS+LIR group (Figures 4(e)–4(g)). The above results suggested that LIR can protect brain injury in mice with FS by reducing mRNA levels and protein expression in the hippocampus of mice with FS.

## 4. Discussion

Chronic FS is a factor that can lead to the onset of epilepsy, and as many as 7% of sick children develop prepubertal epilepsy with severe neuronal injury [19]. The pathogenesis of FS is complex and is a consequence of interactions in immunoinflammatory processes, genetic factors, and activation of cytokine network activation [20]. In clinical studies, it was found to have significantly higher IL-1*β* levels in patients with FS than in fever alone. It was shown that cytokines like IL-6 and anti-inflammatory agents with proinflammatory levels are altered in FS [5]. LIR has the ability to suppress the expression of inflammatory factors, IL-6, TNF-*α*, and nitric oxide (NO) [21, 22]. In this study, 14-day-old male SD mice were collected to establish a model of FS [23].

In patients with type 2 diabetes, GLP-1 increases islet cell proliferation and glucose-dependent insulin production while lowering blood glucose and food consumption [24]. The long-term GLP-1R agonist LIR was widely used in the treatment for DM in clinical [25]. It has been found that GLP-1R is connected with the second messenger pathway of cAMP, which promotes insulin signaling, and expresses in the human and rodent nervous systems, playing a nutritional nerve role [26]. Therefore, we considered that LIR may prevent the development of FS in mice. To explore the association of LIR with FS in mice, the mice were injected with LIR. A lower behavioral score was found in mice with FS after the intervention of LIR, and the seizure latency and seizure duration were significantly shortened. According to these findings that LIR has a therapeutic impact on FS in mice. To further clarify whether LIR affects seizures in mice with FS, mRNA of GLP-1 and GLP-1R in the hippocampus of mice was measured. It was found that GLP-1R was significantly lower in the FS group than the normal groups. But mRNA of GLP-1R in the hippocampus recovered after the intervention of LIR. Thereafter, the expression of GLP-1 and GLP-1R in the hippocampus of mice was detected. The occurrence and development of FS in mice are related with GLP-1. Similarly, a decreased protein expression of GLP-1R was found in the hippocampus with FS. Moreover, after the intervention of LIR, GLP-1R expression recovered in the hippocampus, indicating that the development of FS in mice was related with GLP-1R. Thus, we demonstrated that the expression of GLP-1 and its receptors suppresses the occurrence and development of FS in mice.

RETRACTED

Our current study is the first time the protective impact on LIR on the mice's injured brain with FS. The amount of apoptosis in the hippocampus of mice with FS decreased after giving LIR intervention, and decreased protein expression was found in the hippocampus after the intervention of LIR. It indicates that LIR can reduce the apoptosis of neural cells in the hippocampus of mice with FS. In epilepsy, overexpression of an excitatory glutamate neurotransmitter causes seizure activity by binding to glutamate receptors in the brain [27]. ELISA test found that LIR decreased the glutamate content in the hippocampus of mice with FS. Protein expression of *γ*-aminobutyric acid increased in the hippocampus of mice with FS after the intervention of LIR. The above results showed that LIR can play a protective role against brain injury caused by FS. Our results clearly suggested that LIR can potentially exert a protective effect against brain injury for FS by inhibiting organismic inflammatory factors, like IL-1*β*, IL-6, and TNF-*α*, and results revealed that mRNA and protein of IL-1*β*, IL-6, and TNF-*α* are higher in the hippocampus compared with normal mice. Moreover, mRNA and protein of IL-1*β*, IL-6, and TNF-*α* decreased in the hippocampus after the intervention of LIR.

## 5. Conclusion

Our study found that LIR may protect mice with FS and inhibit or mitigate convulsion-induced brain injury by reducing mRNA levels of inflammatory factors and protein expression in the hippocampus of mice with FS. However, there are still some limitations in our study. We need to collect more data and conduct more detailed and thorough experiments to improve the validness. It provides a new possibility to mitigate and delay the development of FS as well as the prevention and treatment of brain injury caused by FS.

RETRACTED

## Figures and Tables

**Figure 1:** Liraglutide shortened the seizure latency and seizure duration in mice with febrile seizures. (a) Racine grading for behavioral score of mice with FS, to study the correlation of LIR and FS in mice. (b) Examination for seizure latency in mice with FS. (c) Determination for seizures duration in mice with FS. ^∗∗^*P* < 0.01 vs. the control, #*P* < 0.05 vs. FS, and ^∗∗∗^*P* < 0.001 vs. FS, *n* = 10.

**Figure 2:** Levels of GLP-1 and GLP-1R in the hippocampus of mice with febrile seizures. (a) RT-qPCR for mRNA level of GLP-1 in the hippocampus of mice. (b) RT-qPCR for mRNA level of GLP-1R in the mouse hippocampus. (c) Western blot for GLP-1 and GLP-1R protein expressions in the mouse hippocampus. (d) GLP-1 protein expression in the mouse hippocampus. (e) GLP-1R protein expression in the mouse hippocampus. ^∗∗^*P* < 0.01 vs. the control, *^##^P* < 0.01 vs. FS, ^∗∗∗^*P* < 0.001 vs. the control, and ^###^*P* < 0.001 vs. FS, *n* = 10.

**Figure 3:** Effect of LIR on brain injury in mice with febrile seizures (a) TUNEL for apoptosis of hippocampal nerve cells. (b) Protein expression of cleaved-caspase 3 and *γ*-aminobutyric acid (GABA) in the hippocampus of mice. (c) Protein expression of cleaved-caspase 3 in the hippocampus. (d) ELISA for protein expression of glutamate in hippocampus. (e) Protein expression of *γ*-aminobutyric acid (GABA) in the hippocampus of mice. ^∗∗∗^*P* < 0.001 vs. the control, *^###^P* < 0.001 vs. FS, *n* = 10.

**Figure 4:** Expression of inflammatory factors in the hippocampus of mice with febrile seizures. (a) RT-qPCR for mRNA of IL-1*β*. (b) RT-qPCR for mRNA of IL-6. (c) RT-qPCR for mRNA of TNF-*α*. (d) The protein expression of IL-1*β*, IL-6, and TNF-*α*. (e) The protein expression of IL-1*β*. (f) The protein expression of IL-6. (g) The protein expression of TNF-*α*. ^∗∗^*P* < 0.01 vs. the control, *^##^P* < 0.01 vs. FS, *n* = 10. *^###^P* <0.001 vs. the control, *^###^P* < 0.001 vs. FS.

## Data Availability

The datasets used and/or analyzed during the current study are available from the corresponding author on reasonable request.

## References

[1] Asisipo M., Gwladys N. T., Musa M. V. (2020). Effect of a novel prolonged febrile seizure model on GABA associated ion channels. *Metabolic Brain Disease*.

RETRACTED

[2] Yu X., Zhang N., Liu S., Xi Z., Zhang Y. (2018). Polymorphisms in the interleukin-1*β* (IL-1B) and interleukin-1*α* (IL-1A) genes on risk of febrile seizures: a meta-analysis. *Neurological Sciences*.

[3] Garcia-Curran M. M., Hall A. M., Patterson K. P. (2019). Dexamethasone attenuates hyperexcitability provoked by experimental febrile status epilepticus. *Eneuro*.

[4] Warner T. A., Liu Z., Macdonald R. L., Kang J. Q. (2017). Heat induced temperature dysregulation and seizures in Dravet Syndrome/GEFS+ *Gabrg2^+/Q390X^* mice. *Epilepsy Research*.

[5] Gupta S., Aggarwal A., Faridi M. M., Rai G., Das S., Kotru M. (2018). Serum interleukin-6 levels in children with febrile seizures. *Indian Pediatrics*.

[6] Al Morshedy S., Elsaadany H. F., Ibrahim H. E. (2017). Interleukin-1*β* and interleukin-1receptor antagonist polymorphisms in Egyptian children with febrile seizures: a case-control study. *Medicine*.

[7] Ha J., Choi J., Kwon A. (2018). Interleukin-4 and tumor necrosis factor-alpha levels in children with febrile seizures. *Seizure*.

[8] Song C., Wu Y. S., Yang Z. Y. (2019). Astrocyte-conditioned medium protects prefrontal cortical neurons from glutamate-induced cell death by inhibiting TNF-*α* expression. *Neuroimmunomodulation*.

[9] Drucker D. J. (2018). Mechanisms of action and therapeutic application of glucagon-like peptide-1. *Cell Metabolism*.

[10] Knudsen L. B., Lau J. (2019). The discovery and development of liraglutide and semaglutide. *Frontiers in Endocrinology*.

[11] He Z., Gao Y., Lieu L. (2019). Direct and indirect effects of liraglutide on hypothalamic POMC and NPY/AgRP neurons - implications for energy balance and glucose control. *Molecular Metabolism*.

[12] Hussein A. M., Eldosoky M., El-Shafey M. (2019). Effects of GLP-1 receptor activation on a pentylenetetrazole—kindling rat model. *Brain Sciences*.

[13] Zhang Y., Fang J., Feng W., Sun Q., Xu J., Xia Q. (2018). The role of the GLP-1/GLP-1R signaling pathway in regulating seizure susceptibility in rats. *Brain Research Bulletin*.

[14] Wen Y., Wu K., Xie Y., Dan W., Zhan Y., Shi Q. (2019). Inhibitory effects of glucagon-like peptide-1 receptor on epilepsy. *Biochemical and Biophysical Research Communications*.

[15] Anbazhagan A. N., Thaqi M., Priyamvada S. (2017). GLP-1 nanomedicine alleviates gut inflammation. *Nanomedicine*.

[16] Wueest S., Laesser C. I., Böni-Schnetzler M. (2018). IL-6-type cytokine signaling in adipocytes induces intestinal GLP-1 secretion. *Diabetes*.

[17] Patel V. J., Joharapurkar A. A., Kshirsagar S. G. (2018). Coagonist of GLP-1 and glucagon receptor ameliorates development of non-alcoholic fatty liver disease. *Cardiovascular & Hematological Agents in Medicinal Chemistry*.

RETRACTED

[18] Citraro R., Iannone M., Leo A. (2019). Evaluation of the effects of liraglutide on the development of epilepsy and behavioural alterations in two animal models of epileptogenesis. *Brain Research Bulletin*.

[19] Li X., Lin Y., Yao G., Wang Y. (2018). The influence of vaccine on febrile seizure. *Current Neuropharmacology*.

[20] Kothur K., Bandodkar S., Wienholt L. (2019). Etiology is the key determinant of neuroinflammation in epilepsy: elevation of cerebrospinal fluid cytokines and chemokines in febrile infection-related epilepsy syndrome and febrile status epilepticus. *Epilepsia*.

[21] Mei J., Sun J., Wu J., Zheng X. (2019). Liraglutide suppresses TNF-*α*-induced degradation of extracellular matrix in human chondrocytes: a therapeutic implication in osteoarthritis. *American Journal of Translational Research*.

[22] Brock C., Hansen C. S., Karmisholt J. (2019). Liraglutide treatment reduced interleukin-6 in adults with type 1 diabetes but did not improve established autonomic or polyneuropathy. *British Journal of Clinical Pharmacology*.

[23] Sun Q., Zhang Y., Huang J. (2017). DPP4 regulates the inflammatory response in a rat model of febrile seizures. *Bio-medical Materials and Engineering*.

[24] Sharma D., Verma S., Vaidya S., Kalia K., Tiwari V. (2018). Recent updates on GLP-1 agonists: current advancements & challenges. *Biomedicine & Pharmacotherapy*.

[25] Bech E. M., Martos-Maldonado M. C., Wismann P. (2017). Peptide half-life extension: divalent, small-molecule albumin interactions direct the systemic properties of glucagon-like peptide 1 (GLP-1) analogues. *Journal of Medicinal Chemistry*.

[26] Park K. A., Jin Z., Lee J. Y. (2020). Long-lasting exendin-4 fusion protein improves memory deficits in high-fat diet/streptozotocin-induced diabetic mice. *Pharmaceutics*.

[27] Albrecht J., Zielińska M. (2017). Mechanisms of excessive extracellular glutamate accumulation in temporal lobe epilepsy. *Neurochemical Research*.

